# Targeting Mitochondria as Therapeutic Strategy for Metabolic Disorders

**DOI:** 10.1155/2014/604685

**Published:** 2014-03-13

**Authors:** Daniela Sorriento, Antonietta Valeria Pascale, Rosa Finelli, Anna Lisa Carillo, Roberto Annunziata, Bruno Trimarco, Guido Iaccarino

**Affiliations:** ^1^Dipartimento di Scienze Biomediche Avanzate, Università Federico II, Via Pansini 5, 80131 Napoli, Italy; ^2^Dipartimento di Medicina e Chirurgia, Università degli Studi di Salerno, Via Salvador Allende, 84081 Baronissi, Italy; ^3^IRCCS Multimedica, Via Fantoli 16/15, 20138 Milano, Italy

## Abstract

Mitochondria are critical regulator of cell metabolism; thus, mitochondrial dysfunction is associated with many metabolic disorders. Defects in oxidative phosphorylation, ROS production, or mtDNA mutations are the main causes of mitochondrial dysfunction in many pathological conditions such as IR/diabetes, metabolic syndrome, cardiovascular diseases, and cancer. Thus, targeting mitochondria has been proposed as therapeutic approach for these conditions, leading to the development of small molecules to be tested in the clinical scenario. Here we discuss therapeutic interventions to treat mitochondrial dysfunction associated with two major metabolic disorders, metabolic syndrome, and cancer. Finally, novel mechanisms of regulation of mitochondrial function are discussed, which open new scenarios for mitochondria targeting.

## 1. Mitochondria and Cellular Energy

Mitochondria are membrane-bound, cytoplasmic organelles, mainly involved in oxidative energy metabolism by regulating energy homeostasis through the metabolization of nutrients, producing ATP and generating heat [1]. Mitochondria produce more than 90% of our cellular energy by oxidative phosphorylation [2]. Energy production is the result of two metabolic processes—the tricarboxylic acid (TCA) cycle and the electron transport chain (ETC). The TCA cycle uses carbohydrates and fats as substrates for the synthesis of ATP leading to production of the coenzymes NADH and FADH which enter into the ETC in the inner mitochondrion membrane. Mitochondria constantly metabolize oxygen, thereby producing reactive oxygen species (ROS) as a byproduct. Indeed, mitochondria are the most important source of ROS in most mammalian cells. During normal oxidative phosphorylation, in mitochondria, 0.4–4.0% of all oxygen consumed is converted to the superoxide (O_2_^−^) radical [3, 4]. Superoxide is transformed to hydrogen peroxide (H_2_O_2_) by a class of enzymes called superoxide dismutases [5] and then to water by glutathione peroxidase (GPX) or peroxiredoxin III (PRX III) [6]. These organelles have their own ROS scavenging mechanisms that are required for cell survival [7]. Indeed, under normal conditions, the effects of ROS are counteracted by a variety of antioxidants, by both enzymatic and nonenzymatic mechanisms. Oxidative stress is considered as the result of an imbalance of two opposing and antagonistic forces, ROS and antioxidants, in which the effects of ROS are more potent than the compensatory capacity of antioxidants. In turn, excessive ROS production contributes to mitochondrial damage in several conditions and is also important in redox signalling from the organelle to the rest of the cell [8, 9].

## 2. Mitochondrial Dysfunction and Metabolic Disorders

The most important function of mitochondria is the synthesis of ATP by oxidative phosphorylation. Thus, mitochondria generate energy through oxidation of nutrients, such as free fatty acids, to create a proton gradient across the mitochondrial inner membrane used as a source of potential energy to generate ATP, transport substrates or ions, or produce heat [5]. Oxygen radicals are also generated during oxidative phosphorylation which could cause damage of the mitochondrial and cellular DNA, proteins, lipids, and other molecules and leading to oxidative stress and mitochondrial dysfunction. Mitochondrial dysfunction is characterized by inhibition of mitochondrial O_2_ consumption, changes in the mitochondrial membrane potential, and a reduction of ATP levels due to an imbalance between energy intake and expenditure [10]. Damage to mitochondria is primarily caused by ROS generated by the mitochondria themselves [11, 12], in particular by complexes I and III of the electron respiratory chain [13]. Direct damage to mitochondrial proteins decreases their affinity for substrates or coenzymes and, thereby, decreases their function [14]. ROS represented the mechanism of mitochondrial dysfunction during inflammation. Stimulation of cultured cardiac myocytes with tumor necrosis factor (TNF-*α*) or angiotensin II increased ROS generation and myocyte hypertrophy and treatment with antioxidants inhibited both effects [15]. Also TNF-*α* induces mitochondrial dysfunction by reducing complex III activity in the ETC, increasing ROS production, and causing damage to mtDNA [16]. Also the nutrition status and availability of nutrients can cause mitochondrial dysfunction. Indeed, optimal metabolic function of mitochondria depends on the availability of many essential vitamins, minerals, and other metabolites [17, 18]. These micronutrients are critical cofactors that support basic metabolic functions of the mitochondria including ATP and heme synthesis, building electron transport complexes, and detoxification of oxygen. Inadequate amounts of these micronutrients inhibit critical enzymatic activities of the electron transport complexes, thus increasing the production of reactive oxidants and impairing mitochondrial function [17, 18]. For example, several micronutrients (biotin, pantothenate, pyridoxine, riboflavin, copper, iron, and zinc) are required for heme synthesis in mitochondria. A severe deficiency of these micronutrients will cause a deficit of heme and therefore of complex IV, of which heme-a is an essential component [18–20]. The deficits of complex IV result in oxidant leakage, DNA damage, accelerated mitochondrial decay, and cellular aging [18–20].

Mitochondrial dysfunction is closely associated with metabolic disorders [21]. Indeed, it has been demonstrated in various target tissues of metabolic syndrome and insulin resistance including skeletal muscle, liver, fat, heart, and pancreas [22–27]. In skeletal muscle, decreased mitochondrial respiration capacity, reduced ATP production rate, and increased ROS levels lead to reduced fatty acid oxidation and increased cytosolic free acid levels that result in insulin resistance and obesity/diabetes [28–30]. It remains to be established whether mitochondrial dysfunction is the consequence rather than the cause of insulin resistance [31, 32]. Impaired mitochondrial *β*-oxidation is found in patients with nonalcoholic fatty liver disease (NAFLD), a potential cause of hepatic steatosis, and liver injury [33–35], playing an important role in the early stages of liver fibrosis [36]. In adipose tissue, mitochondria provide key intermediates for the synthesis of triglycerides (TGs) and are critical for lipogenesis [37]. Adipose mitochondria are also important for lipolysis through *β*-oxidation of fatty acids, which constitutes an important source of energy for ATP production to supply the energy requirement of the cell. The sirtuins (SIRT) are a class of Nicotinamide Adenine Dinucleotide (NAD)-dependent deacetylase which regulate cellular metabolism. Among them, SIRT3-5 are localized in mitochondria to deacetylate several crucial enzymes involved in mitochondrial functions [38]. SIRT3 deacetylates various key enzymes, such as long-chain acyl-CoA dehydrogenase, leading to an increase of mitochondrial fatty acid oxidation in liver and its deficiency causes metabolic syndrome [39, 40]. In this review, we will deal with the effect of mitochondrial dysfunction in the development of two widespread metabolic disorders, metabolic syndrome and cancer, and the established therapeutic approaches for these conditions.

### 2.1. Mitochondrial Dysfunction in the Metabolic Syndrome

The metabolic syndrome is described as a group of various abnormal metabolic risk factors such as obesity, dyslipidemia, increased blood pressure, increased plasma glucose (prediabetes) levels, prothrombotic condition, and proinflammatory condition [41, 42]. This group of abnormalities recognizes insulin resistance as the intrinsic and common mechanism [41, 43]. Most of the patients with metabolic syndrome gradually develop type 2 diabetes and its complications, like cardiovascular diseases (heart failure, thrombosis, and cardiac arrhythmias). Defective cell metabolism is considered as the main culprits of the syndrome [42] due to the imbalance between nutrient intake and its utilization for energy. Decreased fatty acid oxidation increases the intracellular accumulation of fatty acyl-CoAs and other fat-derived molecules in various organs (adipocytes, skeletal muscle, and liver). This causes the inhibition of insulin signaling leading to hyperinsulinemia which on turn damages various organs in metabolic syndrome [42]. Genetic factors, oxidative stress, mitochondrial biogenesis, and aging affect mitochondrial function, leading to insulin resistance and associated pathological conditions [44–46] (metabolic syndrome, T2DM, and attendant cardiovascular complications) [47–49]. However, it is still not clear whether mitochondrial dysfunction is the primary cause or it is the secondary effect of the metabolic syndrome.

#### 2.1.1. Genetic Factors

Genetic mutations in mitochondrial DNA lead to the so-called mitochondrial diabetes. The most common mutation leading to mitochondrial diabetes is the A3243G mutation in the mitochondrial encoded tRNA (*Leu, UUR*) gene [44, 50]. This mutation leads to impaired synthesis of multiple mitochondrial proteins and overall mitochondrial dysfunction. The A3243G variant of mitochondrial diabetes is characterized by decreased glucose-induced insulin release but not insulin resistance, suggesting that the major pathology occurs within mitochondria of pancreatic *β* cells [44, 50].

#### 2.1.2. Mitochondrial Morphology

Mitochondrial dysfunction could depend on defects in mitochondrial morphology, fission, and fusion. In particular, biopsies of skeletal muscle from subjects with type 2 diabetes and obesity show mitochondria of smaller size and number compared to controls and size appears to correlate with insulin sensitivity [23]. Obesity in both humans and rodents is associated with reduced levels of mitofusin, involved in docking to initiate fusion [51], and polymorphisms of presenillin-associated rhomboid-like (PARL) protein, important for morphologic integrity [52].

#### 2.1.3. Oxidative Phosphorylation and ROS

Impaired mitochondrial biogenesis has been suggested as the cause for reduced mitochondrial number and capacity for oxidative phosphorylation in diabetes [53–55]. Studies of human subjects and rodents provide evidence for impaired oxidative phosphorylation in muscle mitochondria in insulin-resistant states in which there are reduced levels of NADH oxidoreductase and reduced citrate synthase activity [23]. Moreover, in diabetic subjects, there is a decreased mRNA expression of several genes associated with oxidative phosphorylation, including genes coordinately regulated by PGC-1*α* and nuclear respiratory factors [55]. Mitochondrial ROS is involved in both the pathogenesis and long-term complications of diabetes. Indeed, elevated glucose or free fatty acids drive the formation of ROS [56, 57], impairing both *β*-cell insulin release and insulin sensitivity and contributing to the complications of diabetes [6, 58].

#### 2.1.4. Mitochondrial Dysfunction and Insulin Signaling

It has been demonstrated that mitochondrial dysfunction inhibits insulin signaling [59]. Insulin interacts with *α*-subunits of its receptor (IR) on cell membrane. In response to stimuli, tyrosine residues undergo autophosphorylation, and the IR acquires tyrosine kinase activity. This leads to phosphorylation of insulin-receptor substrate-1 (IRS-1), activating a downstream cascade leading to the activation of Akt and translocation of the glucose transporter type 4 (GLUT4) to the cell membrane. GLUT-4 fusion with the membrane results in glucose uptake by facilitated diffusion. Mitochondrial dysfunction is depicted to oppose insulin signaling in two ways: interfering with oxidation of fatty acyl-CoA and consequent accumulation of intracellular lipid and diacylglycerol with consequent activation of protein kinase C [28] and through the generation of ROS [60] (Figure 1). Both processes activate serine kinase reactions, leading to serine phosphorylation of IRS-1, thus interfering with insulin signal transduction. Furthermore, mitochondrial dysfunction seems to play a central role in metabolic and cardiovascular disorders. Cardiovascular diseases, including coronary artery disease, hypertension, heart failure, and stroke, are associated with insulin resistance and diabetes [61, 62]. Free fatty acids (FFAs) contribute to insulin resistance and reduce mitochondrial oxidative capacity, cardiac efficiency, and ATP production and increase myocardial oxygen consumption in obese and insulin-resistant* ob/ob* mice [63]. In addition, intramyocardial lipid accumulation induces lipotoxic injury and cardiac dysfunction, including diastolic dysfunction, left ventricular hypertrophy, and impaired septal contractility in rodent and human obesity [64, 65]. Thus, the reduced mitochondrial oxidative capacity contributes to cardiac dysfunction.

### 2.2. Mitochondrial Dysfunction in Cancer

Several lines of evidence support the hypothesis that cancer is primarily a disease of energy metabolism [66]. Indeed, the mitochondrial dysfunction has been found to be associated with the development of several human cancers [67, 68]. Numerous studies show that tumor mitochondria have impaired morphology and function and are not able to generate normal levels of energy [69–73]. It has been reported that mitochondrial dysfunction in tumors could be caused by inhibitors of mitochondrial electron transport chain [74], pathogenic mutations in mitochondrial DNA (mtDNA), and mutations in nuclear gene coded electron transport chain proteins [75], oncogenic stress, loss of p53 tumor suppressor, and aberrant expression of metabolic enzymes.

#### 2.2.1. Warburg Effect

A prominent alteration in energy metabolism in cancer cells is the increase in aerobic glycolysis, a phenomenon known as the Warburg effect [76, 77]. Recent studies suggest that upregulation of glucose transporters and hexokinases may be involved in promoting the Warburg effect. Elevated expression of glucose transporters (GLUTs) especially GLUT1, which has been correlated with tumor invasiveness and metastasis, is induced by oncogenic transformation caused by c-Myc [78], ras, or scr [79]. C-Myc also activates lactate dehydrogenase A (LDH-A) overexpression, which seems required for c-Myc-mediated transformation [80].

#### 2.2.2. Hypoxia

Mitochondrial dysfunction and hypoxia in the tumor microenvironment are considered as two major factors contributing to the Warburg effect [81–83]. Hypoxia-inducible factor-1 (HIF-1), a transcription factor that regulates the cellular response to hypoxia, induces several genes that mediate tumorigenesis and the development of resistance to chemotherapy [84, 85]. It is known that HIF-1 is a heterodimer that consists of the oxygen sensitive HIF-1*α* subunit and the constitutively expressed HIF-1*β* subunit [86, 87]. Under normoxic conditions, HIF-1*α* is hydroxylated by prolyl hydroxylases on the proline residues in the oxygen-dependent degradation domain [88, 89]. In hypoxic conditions, low oxygen leads to HIF-1*α* stabilization due to the inhibition of prolyl-hydroxylation and subsequent reduction in HIF-1*α* ubiquitination and degradation [89]. Mitochondrial dysfunction promotes cancer cell motility partly through HIF1*α* accumulation mediated via increased production of ROS (Figure 2) [90].

#### 2.2.3. The Tumor Suppressor p53

The tumor suppressor p53 has been shown to be an important molecule that affects glucose metabolism, and loss of p53 function in cancer cells, induced by mitochondrial dysfunction [91], may contribute to the glycolytic phenotype. Wild-type p53 represses GLUT1 and GLUT4 gene transcription, while mutations within the DNA binding domain of p53 impair the repressive effect on GLUT transcription, leading to increased glucose metabolism [92].

#### 2.2.4. ROS Production

Compelling evidence suggests that cancer cells tend to have elevated levels of ROS, compared to the normal cells of the same tissue origins [93]. Cancer cells exhibit increased levels of reactive oxygen species (ROS) partly due to the impaired mitochondrial function [94, 95]. The increased ROS in cancer cells may in turn affect certain redox sensitive molecules and further lead to stimulation of cellular proliferation, cell migration, and invasion, contributing to carcinogenesis [96, 97].

#### 2.2.5. Mitochondrial DNA Mutations

Mitochondrial DNA (mtDNA) mutations correlate with increased ROS levels in solid tumors and leukemia cells [97–99]. Several mtDNA mutations have been identified in various types of human cancer which are present in both the noncoding region and coding regions of the mtDNA [100–104].

#### 2.2.6. Apoptotic Signaling

Proper balance between cell proliferation and cell death is essential to maintain tissue homeostasis, and the failure to eliminate cells by apoptosis may play an important role in carcinogenesis. Abnormal decrease in apoptosis has been considered as a mechanism responsible for the accumulation of cancer cells, especially in certain malignancies such as chronic lymphocytic leukemia [105]. Mitochondria play a pivotal role in regulating apoptosis. Among the important molecules that affect the intrinsic apoptotic pathway through mitochondria, the Bcl-2 family proteins play a major role in cell survival and drug sensitivity since dysregulation of Bcl-2 family is often observed in various types of human cancer, including renal, ovarian, stomach, and brain tumors and leukemia [106–108]. It has been shown that increased expression of prosurvival Bcl-2 homologues [109] or lack of BH3-only protein expression and/or function (e.g., caused by loss of p53) [110] contributed to tumorigenesis and anticancer drug resistance.

## 3. Therapeutic Implications

Giving the main role of mitochondrial dysfunction in the development of several metabolic disorders, new therapeutic strategies have been developed during the last years to regulate mitochondrial function and biogenesis. These approaches could be useful to decrease insulin action and pancreatic beta-cell production, lipid accumulation in liver, skeletal muscle impairments, endothelial-mediated vasorelaxation, and both systolic and diastolic myocardial function. Pharmacologic interventions are focused on mechanisms regulating mitochondrial biogenesis, ROS, and respiration thus to restore mitochondrial function as well as mitochondrial ROS production.

### 3.1. Pharmacological Interventions

Newer pharmacologic approaches have been proposed to improve mitochondrial function. Resveratrol, an ingredient of red wines, is a polyphenolic SIRT1 activator that, like calorie restriction, has antiaging effects in lower organisms [111], reduces signs of aging in mice, and extends survival [112]. In mice, resveratrol improves insulin resistance, protects against diet-induced obesity, induces genes for oxidative phosphorylation, and activates PGC-1*α* [113]. Other related small molecules are more potent than resveratrol to enhance the action of SIRT1 on substrates for deacetylation [114]. Similar to resveratrol, these compounds bind directly to the SIRT1-acetylated peptide complex at the same site and lower the *K*_*m*_ for peptide substrate resulting in a more productive catalytic complex [114]. Other potential targets for pharmacologic manipulation include AMPK [115], which enhances both glucose and fat oxidation [116, 117], pyruvate dehydrogenase [118], or the various shuttle mechanisms regulating uptake of TCA intermediates. Moreover, as recently showed [119], mitochondria targeted antioxidants may alter intact-cell fuel selectivity. Various vitamins and chemical compounds with antioxidant properties have been developed, including coenzyme Q [120], vitamin E [121], a-lipoic acid [122], N-acetylcysteine (NAC) [123], vitamin C, and inducers of heme oxygenase [124], which are able to reduce ROS production. Successively, antioxidant compounds specifically targeted to mitochondria have been synthesized, incorporating ubiquinone (mitoQ) or vitamin E (mitoVit E) [125]. Oral administration of mitoQ (500 mM in drinking water administered ad libitum) to normal male rats protected heart muscle function, prevented myocardial cell death, and improved the respiratory-control ratio (state 3 to state 4 respiration) in rats subject to ischemia/reperfusion injury [126]. Mitochondrial-targeted antioxidants protected Friedreich ataxia fibroblasts, in which glutathione synthesis was blocked, from oxidative stress [127] and reduced telomere shortening [128]. In bovine aortic endothelial cells, mitoQ reduced oxidative damage in cells stressed by 25 mM glucose and glucose oxidase [129]. Moreover, mitoQ also reduced ROS and reduced activation of the mitogen-activated protein kinase, p42-ERK2, in endothelial cells after hypoxic stress [130].

### 3.2. Exercise and Diet

Lifestyle modification, including exercise and diet, decreases the risk for developing type 2 diabetes [131], whereas physical activity improves glucose tolerance [132]. Exercise offers several benefits, including increased electron-transport activity in muscle, stimulation of mitochondrial biogenesis through effects on PGC-1*α*, and improved sensitivity to insulin [133, 134]. Moreover, it has been shown that it also activates AMPK, which improves both glucose and fat oxidation [133].

### 3.3. Therapeutic Approaches for Cancer

The primary strategic problem in cancer therapy is how to selectively activate apoptosis in transformed cells. Despite the heterogeneity of tumors and a consequent need of an individual approach for anticancer treatment, many tumor cells demonstrate enhanced uptake and utilization of glucose which leads to the stabilization of the mitochondria and an increased resistance to outer mitochondrial membrane (OMM) permeabilization and apoptotic cell death. Thus, a successful therapy should be based on the activation of apoptotic pathways, which are suppressed in tumor cells. Targeting mitochondria might be a promising strategy to increase the sensitivity of tumor cells to apoptotic stimuli [135, 136]. Suppression of pyruvate dehydrogenase kinase (PDK1) and LDH activities decreased mitochondrial membrane potential and increased mitochondrial production of ROS in cancer cells, but not in normal cells [137]. Similarly, overexpression of frataxin, a protein associated with Friedreich ataxia, stimulated oxidative metabolism and elevated mitochondrial membrane potential and ATP content in several colon cancer cell lines [138]. The Bcl-2 homology 3 (BH3) domain is crucial for the death-inducing and dimerization properties of proapoptotic members of the Bcl-2 protein family. It has been demonstrated that synthetic peptides corresponding to the BH3 domain of Bak bind to Bcl-x_L_, antagonize its anti-apoptotic function, and rapidly induce apoptosis when delivered into intact cells via fusion to the Antennapedia homeoprotein internalization domain [139]. Treatment of HeLa cells with the Antennapedia-BH3 fusion peptide resulted in peptide internalization and induction of apoptosis within 2-3 hours [139].

## 4. Conclusions and Perspectives

Mitochondria are vital for cell function and survival; thus, it is not surprising that the loss of integrity of these organelles is associated with several pathological conditions. To date, great advances have been made to improve the knowledge of the link between mitochondrial dysfunction and metabolic diseases and different therapeutic approaches have been developed to reestablish normal function of the organelles and restore cellular homeostasis. However, an important question remains to be answered: is mitochondrial dysfunction a contributing factor or a consequence of metabolic diseases? Further studies are needed to solve this issue and to provide new insights for the development of specific and effective therapeutic treatments of metabolic diseases.

## Figures and Tables

**Figure 1:** Mitochondrial dysfunction regulates insulin signaling. Insulin interacts with *α*-subunits of its receptor (IR) on cell membrane. In response to stimuli, tyrosine residues undergo autophosphorylation, and the IR phosphorylates the insulin-receptor substrate-1 (IRS-1) in serine residues, activating Akt, with phosphorylation of the type 4 glucose transporter (GLUT4) to the cell membrane and facilitation of glucose uptake. Mitochondrial dysfunction inhibits insulin signaling, leading to insulin resistance, by (1) interfering with oxidation of fatty acyl-CoA and consequent accumulation of diacylglycerol, with consequent activation of protein kinase C and phosphorylation of IRS-1 in tyrosine residues preventing its activation, and (2) through the generation of ROS, which inhibits IRS phosphorylation in serine residues.

**Figure 2:** Mitochondrial dysfunction and hypoxia in cancer. Schematic representation of the role of mitochondrial dysfunction in tumorigenesis. Damaged mitochondria release ROS which on turn activates HIF1*α*. Finally, HIF1*α* activates the tumorigenic hypoxia pathway by initiating transcription of genes involved in glucose metabolism, angiogenesis, and survival.
